The article "Observation on the Efficacy of Ginkgo Ketone Ester Drop Pill in Improving Hypertension Combined with Carotid Atherosclerotic Plaque" was published in 2022. Journal: Emerg Med Int.

# Observation on the Efficacy of *Ginkgo* Ketone Ester Drop Pill in Improving Hypertension Combined with Carotid Atherosclerotic Plaque

**DOI:** 10.1155/2022/8650537

**Published:** 2022-06-30

**Authors:** Jie Zhang, Yingli Ma

**Affiliations:** ^1^Ningbo Women's and Children's Hospital, Ningbo 315000, Zhejiang, China; ^2^Department of Neurology, Ningbo Hospital of Traditional Chinese Medicine, Ningbo 315000, Zhejiang, China

## Abstract

**Purpose:**

To observe and analyze the efficacy of *Ginkgo* ketone ester drop pill intervention in patients with hypertension combined with carotid atherosclerotic plaque.

**Methods:**

The subjects were 300 patients with hypertension complicated with carotid atherosclerotic plaque treated in our hospital from January 2019 to September 2021. The grouping was done by the random number table method and 300 patients were divided equally into 2 groups. One group was treated with Western medicine alone (clopidogrel sulfate tablets, phenyl amlodipine tablets, irbesartan tablets, and resorvastatin) as the Western medicine group (WM group, *n* = 150), and one group was added to this intervention with *Ginkgo* ketone ester drop pill as the Chinese medicine group (CM group, *n* = 150). The observation indexes were the improvement of blood pressure (systolic blood pressure (SBP) and diastolic blood pressure (DBP)), blood lipids (low-density lipoprotein cholesterol (LDL-C), high-density lipoprotein cholesterol (HDL-C), triglyceride (TG), and total cholesterol (TC)), vascular endothelial function (nitric oxide (NO) and endothelin-1 (ET-1)), inflammatory factors (C-reactive protein (CRP) and interleukin-6 (IL-6)), plaque (intimal medial thickness (IMT) of carotid artery and plaque area), and efficacy after intervention and adverse effects during intervention in both groups.

**Results:**

After intervention, SBP, DBP, LDL-C, TG, and TC levels were lower and HDL-C levels were higher in both groups than before intervention in the same group, and both CM groups improved significantly compared with the WM group (*P* < 0.05). After intervention, NO levels were higher and ET-1 levels were lower in both groups than before the intervention in the same group, and both CM groups improved significantly compared with the WM group (*P* < 0.05). After intervention, CRP and IL-6 levels were lower in both groups than before intervention in the same group, and both CM groups improved significantly compared with the WM group (*P* < 0.05). After intervention, IMT and plaque area were lower in both groups than before intervention in the same group and both CM groups improved significantly compared with the WM group (*P* < 0.05). The total effective number of the CM group was better than the WM group (*P* < 0.05), and there was no significant difference in the adverse reactions number in both groups (*P* > 0.05).

The article "Observation on the Efficacy of Ginkgo Ketone Ester Drop Pill in Improving Hypertension Combined with Carotid Atherosclerotic Plaque" was published in 2022. Journal: Emerg Med Int.

**Conclusions:**

The treatment of hypertension combined with carotid atherosclerotic plaque with *Ginkgo* ketone ester drop pill helps to improve the blood pressure, blood lipid, and vascular endothelial function of patients and helps to inhibit the inflammation level and atherosclerotic plaque of patients, with significant efficacy and no significant adverse effects in patients, which is worthy of clinical promotion.

## 1. Introduction

Hypertension is a group of cardiovascular syndromes caused by a combination of genetic, environmental, and other factors in a continuous state of progression, of which primary hypertension is more common, accounting for about 90% of clinical cases [1]. The disease has an insidious onset and mild symptoms, but if blood pressure is chronically elevated, it can cause changes in the function and structure of the heart and blood vessels [2]. The latter is mainly reflected in the long-term increase in blood pressure that increases the impact of blood on the arterial wall, which results in impaired intima and endothelial function, leading to the deposition of lipids and inflammatory factors such as interleukin (IL) in blood in the vessel wall, which eventually induces the formation of atherosclerosis (AS) and its atheromatous plaque, one of the main risk factors for the formation of ischemic cerebral infarction [3–5]. Conversely, the occurrence of AS causes a decrease in the diastolic function of the blood vessels, an increase in the sclerosis of the vessel walls, and a consequent increase in blood pressure [6]. The two are mutually beneficial, forming a vicious circle and increasing the risk of cardiovascular disease.

Preliminary pharmacological studies have shown that the combination of platelet aggregation inhibitors, calcium antagonists, angiotensin-converting enzyme inhibitors, and statins for the treatment of hypertension combined with carotid atherosclerosis has additive effects in regulating blood pressure and lipids and stabilizing atheromatous plaques [7–9]. In addition, as a classical therapeutic drug for cardiovascular and cerebrovascular diseases in Chinese medicine, *Ginkgo biloba* ketone ester also has a good regulatory effect on blood lipids and vascular endothelial cell function. However, there are no detailed clinical reports on whether the combination of the two can produce good synergistic effects and whether the adverse effects are superimposed. This study makes preliminary observation and analysis in order to provide more efficient treatment for this kind of patients. The report is as follows.

The article "Observation on the Efficacy of Ginkgo Ketone Ester Drop Pill in Improving Hypertension Combined with Carotid Atherosclerotic Plaque" was published in 2022. Journal: Emerg Med Int.

## 2. Materials and Methods

### 2.1. General Information

The subjects were 300 patients with hypertension complicated with carotid atherosclerotic plaque treated in our hospital from January 2019 to September 2021. The grouping was done by the random number table method and 300 patients were divided equally into 2 groups. One group was treated with Western medicine alone (clopidogrel sulfate tablets, phenyl amlodipine tablets, irbesartan tablets, and resorvastatin) as the Western medicine group (WM group, *n* = 150), and one group was added to this intervention with *Ginkgo* ketone ester drop pill as the Chinese medicine group (CM group, *n* = 150). The difference in general information in both groups was not statistically significant (*P* > 0.05) and was comparable. The details are given in Table 1.

### 2.2. Inclusion Criteria

The inclusion criteria were as follows: meet the CHEP (Canadian Hypertension Education Program) hypertension guidelines [10] for the diagnosis of hypertension: systolic blood pressure (SBP) ≥ 140 mm·Hg and/or diastolic blood pressure (DBP) ≥ 90 mm·Hg (1 mm·Hg = 0.133 kPa); meet the ACC (American College of Cardiology/AHA (American Heart Association) guidelines for secondary prevention of patients with coronary artery disease and other atherosclerotic vascular disease [11] for the diagnosis of carotid atherosclerosis: intimal medial thickness (IMT) of carotid arteries ≥1.3 mm suggesting plaque formation; age of onset 40–75 years; carotid color Doppler ultrasound showed atheromatous plaque at any of the carotid bifurcation, the distal bilateral common carotid arteries, or the beginning of the internal carotid artery; primary hypertension; and those who had signed written informed consent.

### 2.3. Exclusion Criteria

The exclusion criteria were as follows: secondary hypertension; persons with severe coagulation disorders, autoimmune diseases, hyperuricemia, diabetes mellitus, hyperlipidemia, and hepatic and renal insufficiency; persons with contraindications to the use of drugs in this study; persons with malignant tumors; persons with acute and chronic inflammation; pregnant and lactating women; persons with the history of stroke and serious heart disease; and persons with mental disorders that prevent them from communicating properly.

### 2.4. Medication Regimen

The WM group was intervened with Western medicine intervention alone: i.e., mild hypertension was treated with clopidogrel sulfate tablets (Sanofi (Hangzhou) Pharmaceutical Co., Ltd., National Drug Administration J20130083, 75 mg *x* 7 slices) 75 mg + phenyl amlodipine tablets (Guangdong Pidi Pharmaceutical Co., Ltd., National Drug Administration H20057316, 5 mg *x* 14 slices) 5 mg + resorvastatin (AstraZeneca Pharmaceutical Co., Ltd., National Drug Administration J20120006, 10 mg/slice) 10 mg, 1 time/day. Moderate hypertension was treated with irbesartan tablets (Yangtze River Pharmaceutical Group Beijing Haiyan Pharmaceutical Co., Ltd., National Drug Administration H20100164, 75 mg *x* 12 slices) 75 mg in addition to mild hypertension, 1 time/day. Severe hypertension was treated with irbesartan tablets 150 mg in addition to mild hypertension, 1 time/day.

The article "Observation on the Efficacy of Ginkgo Ketone Ester Drop Pill in Improving Hypertension Combined with Carotid Atherosclerotic Plaque" was published in 2022. Journal: Emerg Med Int.

The CM group was intervened with *Ginkgo* ketone ester drop pill in addition to the WM group, *Ginkgo* ketone ester drop pill (Shanxi Qianhui Pharmaceutical, National Drug Administration Z20050220, 120 pills/bottle), each time 5 pills, 3 times/day. 4 weeks as a course of treatment, both groups continued treatment for 3 courses.

### 2.5. Observation Index

Before and after intervention, 10 ml of fasting elbow venous blood was drawn from both groups in the early morning, centrifuged at 2 000 r/min for 30 min at high speed and low temperature, and serum was stored in a refrigerator at −20°C (Table 2).

1. Blood pressure: before and after intervention, SBP and DBP of both groups were measured by the mercury sphygmomanometer, and the examination method was to measure once every 5 min interval and three times continuously, and the average value was taken as the final result.
2. Blood lipids: before and after intervention, two groups of low-density lipoprotein cholesterol (LDL-C) and high-density lipoprotein cholesterol (HDL-C) were detected by the direct homogeneous method, and the kits were purchased from Changchun Huili Biotechnology Co. Ltd.; two groups of triacylglyceride (TG) were detected by the glycerol phosphate oxidase-peroxidase coupling method, and the kit was purchased from Zhejiang Taisite Biotechnology Co. Ltd.; two groups of total cholesterol (TC) were detected by high performance liquid chromatography, and the instrument was purchased from Shanghai Hegong Scientific Instrument Co. Ltd., and the instrument model was Vertex Sti P5000. Among them, LDL-C ≥ 3.64 mmol/L, TG > 1.70 mmol/L, and TC ≥ 5.72 mmol/L indicated an increase and HDL-C < 0.91 mmol/L indicated a decrease.
3. Vascular endothelial function: before and after intervention, two groups of nitric oxide (NO) and endothelin-1 (ET-1) levels were detected by enzyme-linked immunosorbent assay (ELISA), and the kit was purchased from Tianjin Sairuida Bioengineering Co. Ltd.
4. Inflammatory factors: before and after intervention, two groups of C-reactive protein (CRP) levels were detected by immune scattering turbidimetry, and the kit was purchased from Nanjing Jiancheng Bioengineering Institute; two groups of interleukin-6 (IL-6) levels were detected by ELISA, and the kit was purchased from Guangdong Hongye Antibody Technology Co. Ltd.
5. Plaque condition: before and after intervention, the IMT and plaque area of both groups were detected by using the American HP-8500 color Doppler ultrasound diagnostic instrument. IMT measurement method: patients were placed in a supine position, the anterior part of the neck was exposed, and the IMT of the carotid bifurcation, the distal bilateral common carotid arteries, and the beginning of the internal carotid artery were detected at a probe frequency of 7.5 MHz on the near skin side. IMT <1.0 mm indicated normal, ≥1.0 mm indicated thickening, and ≥1.3 mm indicated plaque formation.
6. Clinical efficacy: refer to the Guiding Principles for Clinical Research on New Chinese Medicines [12] to develop efficacy determination criteria for more details.
7. Adverse effects: during intervention, the occurrence of dizziness, diarrhea, poor appetite and indigestion, and others were recorded in both groups.

The article "Observation on the Efficacy of Ginkgo Ketone Ester Drop Pill in Improving Hypertension Combined with Carotid Atherosclerotic Plaque" was published in 2022. Journal: Emerg Med Int.

### 2.6. Statistical Methods

Data were processed using the SPSS 22.0 software. The count data were expressed as (%) and the *χ*^2^ test was taken. The measurement data were expressed as ($\bar{x}$ ± *s*), and the *t*-test was taken. Statistically significant differences were expressed as *P* < 0.05.

## 3. Results

### 3.1. Comparison of SBP and DBP Levels in Both Groups

After intervention, SBP and DBP levels were lower in both groups than before intervention in the same group, and both CM groups improved significantly (*P* < 0.05) than in the WM group (Figure 1).

### 3.2. Comparison of LDL-C, HDL-C, TG, and TC Levels in Both Groups

After intervention, LDL-C, TG, and TC levels were lower and HDL-C levels were higher in both groups than before intervention in the same group, and both CM groups improved significantly (*P* < 0.05) than the WM group (Figure 2).

### 3.3. Comparison of NO and ET-1 Levels in Both Groups

After intervention, NO levels were higher and ET-1 levels were lower in both groups than before intervention in the same group, and both CM groups improved significantly (*P* < 0.05) than the WM group (Figure 3).

### 3.4. Comparison of CRP and IL-6 Levels in Both Groups

After intervention, CRP and IL-6 levels were lower in both groups than before intervention in the same group, and both CM groups improved significantly (*P* < 0.05) than the WM group (Figure 4).

### 3.5. Comparison of IMT and Plaque Area in Both Groups

After intervention, IMT and plaque area were lower in both groups than before intervention in the same group, and both CM groups improved significantly (*P* < 0.05) than the WM group (Figure 5).

The article "Observation on the Efficacy of Ginkgo Ketone Ester Drop Pill in Improving Hypertension Combined with Carotid Atherosclerotic Plaque" was published in 2022. Journal: Emerg Med Int.

### 3.6. Comparison of Clinical Efficacy and Adverse Effects in Two Groups

After intervention, the total effective number was better in the CM group than in the WM group (*P* < 0.05) (Figure 6). During intervention, there was no significant difference (*P* > 0.05) in adverse reactions number in both groups (Figure 7).

## 4. Discussion

Hypertension is a common clinical chronic disease, and the rise of peripheral blood pressure is its main characteristic, which is also the main cause of carotid atherosclerosis and its plaque formation. Patients may often see clinical manifestations such as dizziness, headache, palpitations, insomnia, blurred vision, temporal pulsation sensation, and in severe cases, cerebral infarction, resulting in hemiparesis and limited mobility of one limb [13–15]. Moreover, when hypertension and carotid atherosclerotic plaque coexist, patients have a higher risk of cardiovascular and cerebrovascular events, while the treatment methods of improving lipid metabolism disorder and vascular endothelial function and stabilizing the nature of atherosclerotic plaque may prevent the occurrence of cardiovascular and cerebrovascular diseases [16].

Hypertension patients' blood pressure increases, vascular endothelial function is damaged, the balance of vascular SBP and DBP is destroyed, and the permeability of endothelial cells is increased, resulting in the decrease of NO, the increase of ET-1, platelet aggregation, the production of inflammatory factors, and finally the generation of AS. Clopidogrel sulfate tablet is a platelet aggregation inhibitor, which can selectively inhibit the binding of platelet membrane adenosine diphosphate to platelet receptor to inhibit platelet aggregation caused by arterial intimal damage, so as to block microthrombotic formation and prevent AS [17]. Phenyl amlodipine tablet is a calcium antagonist antihypertensive drug, and irbesartan tablet is an angiotensin receptor blocker (ARB) antihypertensive drug. If necessary, the combined application of the two can improve the curative effect and reduce adverse reactions [18]. Rosuvastatin is a selective HMG CoA reductase inhibitor. Its main action site is the liver, the target organ for reducing cholesterol [19].

According to the theory of traditional Chinese medicine, hypertension complicated with carotid atherosclerotic plaque belongs to the categories of “headwind,” “stroke,” and “vertigo.” The pathogenesis is the deficiency of fundamental and the excess of incidental, the deficiency of healthy Qi, and the excess of evil Qi, deficiency intermingled with excess. Deficiency lies in Yin deficiency of internal organs, excess lies in blood stasis and phlegm turbidity, and developing into paralysis obstruction. The treatment should adopt the method of promoting blood circulation, removing blood stasis, and dredging collaterals. This study observed and analyzed the effect of *Ginkgo* ketone ester drop pill on patients with hypertension complicated with carotid atherosclerotic plaque. The results show that after intervention, SBP, DBP, LDL-C, TG, TC, and ET-1 levels in both groups were lower and HDL-C and NO levels were higher than before intervention in the same group, and both CM groups improved significantly (*P* < 0.05) than the WM group. It was suggested that the addition of *Ginkgo* ketone ester drop pill to conventional Western medicine treatment for hypertension combined with carotid atherosclerotic plaque could significantly regulate the patients' blood pressure and lipid levels and improve the endothelial function of blood vessels. *Ginkgo* ketone ester drop pill are an extract of *Ginkgo biloba*, which belongs to the fifth generation of *Ginkgo biloba* preparations. Its active ingredients are mainly *Ginkgo* flavonoids and ginkgolide, while the content of ginkgolic acid is low. In terms of the mechanism of action in modern medicine, it is directly absorbed into blood through oral mucosa, avoiding the first-pass effect of the drug, so it has the advantages of better efficacy in activating blood circulation and removing blood stasis, faster onset of action, and higher safety. It not only improves vascular permeability, dilates blood vessels, and increases cerebral blood flow, thereby lowering blood pressure, but also specifically antagonizes platelet-activating factor (PAF), protects the corresponding target organs, reduces blood viscosity, improves microvascular function, and plays an anti-AS role [20, 21]. In traditional Chinese medicine, *Ginkgo* is a good medicine for promoting blood circulation and removing blood stasis, which has the effects of promoting blood circulation and removing blood stasis, dredging veins, and relaxing collaterals. Previous studies have shown that the reason why *Ginkgo biloba* ketone ester dropping pills can effectively reduce cardiovascular and cerebrovascular events may also be related to its effect of inhibiting oxidative stress response and scavenging free radicals [22].

The article "Observation on the Efficacy of Ginkgo Ketone Ester Drop Pill in Improving Hypertension Combined with Carotid Atherosclerotic Plaque" was published in 2022. Journal: Emerg Med Int.

AS is mostly triggered initially by hyperlipidemia. Leukocytes adhere to the vessel lining and then move to the subendothelium to phagocytose liposomes, which eventually transform into foam cells and destroy the vascular endothelium on the basis of this chronic inflammatory pathological response and activate the platelet system, leading to luminal narrowing, obstruction, and plaque formation [23]. With the increasing volume of plaque, it causes vascular obstruction and blood circulation obstruction, resulting in serious cardiovascular and cerebrovascular diseases. CRP is an acute phase reactive inflammatory protein, and its expression level is positively correlated with plaque area [22]. IL-6 is a marker of progressive AS, which can induce or aggravate cardiovascular disease by promoting plaque growth and is an independent predictor of plaque progression [24]. The location of carotid artery is relatively shallow and easy to measure. Measuring IMT can reflect the situation of systemic AS and is an independent predictor of cardiovascular and cerebrovascular events [25]. In the results of this study, after intervention, CRP and IL-6 levels and IMT and plaque area were lower in both groups than before intervention in the same group, and both CM groups improved significantly (*P* < 0.05) than the WM group. It is suggested that the effective mechanism of *Ginkgo* ketone ester drop pill in the treatment of hypertension complicated with carotid atherosclerotic plaque may also be related to its inhibition of inflammatory response. The results also showed that the total effective number was better in the CM group than in the WM group (*P* < 0.05), and there was no significant difference (*P* > 0.05) in adverse reactions number in both groups. It shows that *Ginkgo* ketone ester drop pill is effective and safe in the treatment of hypertension complicated with carotid atherosclerotic plaque. Analyzing the reason, it may be because the toxic component of *Ginkgo biloba* ketone ester preparation is mainly ginkgolic acid, and the process of domestic *Ginkgo biloba* ketone ester has become mature, and the content of ginkgolic acid can be controlled below 5 *μ*g/*g*, so its adverse reactions are less.

In short, the treatment of hypertension combined with carotid atherosclerotic plaque with *Ginkgo* ketone ester drop pill helps to improve the blood pressure, blood lipid, and vascular endothelial function of patients and helps to inhibit the inflammation level and atherosclerotic plaque of patients, with significant efficacy and no significant adverse effects in patients, which is worthy of clinical promotion. The shortcomings of this study include the short follow-up observation of patients and the relatively superficial studies related to adverse drug reactions; in the future, we will extend the follow-up period for further studies and pay attention to the observation of adverse drug reactions.

## Figures and Tables

**Figure 1:** Comparison of SBP and DBP levels in both groups. (a) SBP level. (b) DBP levels. Compared with the same group before intervention, ^∧^*P* < 0.05; compared with the WM group after intervention, ^*∗*^*P* < 0.05.

The article "Observation on the Efficacy of Ginkgo Ketone Ester Drop Pill in Improving Hypertension Combined with Carotid Atherosclerotic Plaque" was published in 2022. Journal: Emerg Med Int.

**Figure 2:** Comparison of LDL-C, HDL-C, TG, and TC levels in both groups. (a) LDL-C levels. (b) HDL-C levels. (c) TG level. (d) TC levels. Compared with the same group before intervention, ^∧^*P* < 0.05; compared with the WM group after intervention, ^*∗*^*P* < 0.05.

**Figure 3:** Comparison of NO and ET-1 levels in both groups. (a) NO levels. (b) ET-1 levels. Compared with the same group before intervention, ^∧^*P* < 0.05; compared with the WM group after intervention, ^*∗*^*P* < 0.05.

**Figure 4:** Comparison of CRP and IL-6 levels in both groups. (a) CRP levels. (b) IL-6 levels. Compared with the same group before intervention, ^∧^*P* < 0.05; compared with the WM group after intervention, ^*∗*^*P* < 0.05.

**Figure 5:** Comparison of IMT and plaque area in both groups. (a) IMT. (b) Plaque area. Compared with the same group before intervention, ^∧^*P* < 0.05; compared with the WM group after intervention, ^*∗*^*P* < 0.05.

**Figure 6:** Comparison of clinical efficacy in two groups. Comparison between groups, ^∧^*P* < 0.05.

**Figure 7:** Comparison of adverse effects in two groups.

**Table 1:** Comparison of general information for both groups.

Indicators	WM group (*n* = 150)	CM group (*n* = 150)	*t*/*χ*^2^	*P*
Age (years old)	58.21 ± 7.09	58.91 ± 7.25	0.845	0.399
Height (cm)	166.89 ± 5.84	166.93 ± 5.46	0.061	0.951
Weight (case)	70.14 ± 6.48	69.25 ± 7.10	1.134	0.258
Course of hypertension (years)	5.71 ± 1.23	5.56 ± 1.26	1.043	0.298
Male (case)	89 (59.33)	94 (62.67)	0.350	0.554
Stroke history (case)	40 (26.67)	36 (24.00)	0.282	0.595

**Table 2:** Criteria for determining efficacy.

Criteria	Efficacy index	Symptoms and signs	Blood pressure
Ineffective	<30%	None improved	SBP and DBP are not decreasing and not trending downward
Effective	≥30%	All significantly better	SBP decreased <20 mm·Hg, DBP decreased <10 mm·Hg
Significantly effective	≥70%	All largely disappeared	SBP decreased ≥20 mm·Hg, DBP decreased ≥10 mm·Hg
Total effective number = significantly effective number + effective number			

Efficacy = (postintervention−preintervention)/preintervention score × 100%.

## Data Availability

The datas used and analyzed during the current study are available from the corresponding author upon request.
